# Operational Scheduling of Behind-the-Meter Storage Systems Based on Multiple Nonstationary Decomposition and Deep Convolutional Neural Network for Price Forecasting

**DOI:** 10.1155/2022/9326856

**Published:** 2022-02-21

**Authors:** Zhuofu Deng, Xianglong Qi, Tengteng Xu, Yingnan Zheng

**Affiliations:** ^1^Software College, Northeastern University, Shenyang, Liaoning 110 169, China; ^2^Liaoning Huading Technology Co.,Ltd., Shenyang, Liaoning 110 167, China

## Abstract

In the competitive electricity market, electricity price reflects the relationship between power supply and demand and plays an important role in the strategic behavior of market players. With the development of energy storage systems after watt-hour meter, accurate price prediction becomes more and more crucial in the energy management and control of energy storage systems. Due to the great uncertainty of electricity price, the performance of the general electricity price forecasting models is not satisfactory to be adopted in practice. Therefore, in this paper, we propose a novel electricity price forecasting strategy applied in optimization for the scheduling of battery energy storage systems. At first, multiple nonstationary decompositions are presented to extract the most significant components in price series, which express remarkably discriminative features in price fluctuation for regression prediction. In addition, all extracted components are delivered to a devised deep convolution neural network with multiscale dilated kernels for multistep price forecasting. At last, more advanced price fluctuation detection serves the optimized operation of the battery energy storage system within Ontario grid-connected microgrids. Sufficient ablation studies showed that our proposed price forecasting strategy provides predominant performances compared with the state-of-the-art methods and implies a promising prospect in economic benefits of battery energy storage systems.

## 1. Introduction

Over the last decades, the power grid operations are provided more and more pressure when electricity consumption increases sharply. In addition, the use of fossil fuels for electricity generation brings more environmental concerns, especially in peak hours when the grid is running inconsistent with its operation limits and becoming more delicate. The behind-the-meter (BTM) energy storage system is able to unify communicating, automatic control, and sensor technologies to reshape the electricity consumption activity efficiently and has been widely applied for both the grid-connected and islanded operation of microgrids [1]. Because of irregularities within generation sections, important modules of BTM are decided on the orchestration of loads through efficient optimization. Moreover, BTM systems aim to offer better electricity consumption services for users based on their response demand by connecting to household terminals [2]. Consequently, tasks of BTM operating systems explore more effective approaches to reduce operation costs, improve energy efficiency, and balance requirements of demand and supply [3]. In the attractive electricity market, the price of electricity always fluctuates with changes in the supply and demand of the market. At this time, the BTM system can be employed to control the peak price for large customers [4], who expect to purchase electricity at a relatively lower price and deliver it to end users at a higher price. Therefore, in this paper, we give most attention to a multistep electricity price forecasting method that benefits optimization of scheduling in BESS for economic objectives.

Approaches of electricity price forecasting give more significance in practice since they will produce profits in areas of energy management, demand response (DR), grid operations, etc. [5]. In a comparison of load forecasting in the short term, the uncertainty of electricity price is more complicated, which shows great nonlinear relationships within electricity profiles. Electricity sellers and buyers express their requirements with bids in the electricity trading market, and prices of these bids are resolved by all market players forming a uniform market clearing price (MCP) [6]. BTM Battery Energy Storage Systems (BESS) is supposed to serve a large group of customers generally and operate in the local grid considering more comprehensive factors. For example, in Ontario, BESS could not only offer electricity for local consumers satisfying their real-time needs but also deliver redundant powers to upper-level grid buyers for profitable sales.

In general, most of the research on price forecasting focuses on the short term, which has close relationships with energy management and real-time scheduling of BESS. Research is grouped into three classes: single point, probability, and multithreshold forecasting [7]. Point prediction offers only one simple value [8], and in contrast, probability prediction provides quantile intervals to quantify uncertainties for short-term price fluctuation [9, 10]. In practice, the target of electricity price forecasting has no exact requirement to point predication, but prespecified price thresholds served in the process of decision instead, such as DR, which gives more crucial significance to commercial decisions in the electricity market [11–13].

Specifically, electricity price forecasting cannot fulfill all requirements of optimization in BESS completely. If more advanced price spike detection was given, the economic savings of BESS should be given more power using advanced statistical or machine learning models. These popular models rely on the historical dataset of price changes and additional factors such as holidays, temperature trends, periodical characters, and DR pLans and extract excellent hand-crafted features for deep analysis. The Autoregressive (AR) model has been widely introduced in time sequence analysis using a statistical algorithm, which shows excellent capability in tracking price fluctuations. A recursive dynamic factor analysis (RDFA) is proposed by Wu et al. [14], unifying a Kalman Filter model to demonstrate an advanced strategy that outperformed the state-of-the-art research for price spike forecasting. Amjady and Keynia [15] presented a new electricity price peak occurrence and peak prediction strategy, which is based on information theory and includes a new closed-loop prediction mechanism. Christensen et al. [16] set up a nonlinear variant of the AR conditional hazard model to simulate the electricity price trading process for spike detection in the Australian electricity market. Zhao et al. [17] devised an innovative feature selector to discriminate specific attributes relative to emergences of spike based on a data mining approach. Fragkioudaki et al. [18] and Lu et al. [19] similarly trained a classifier via hand-crafted features derived from electricity price occurrences. Although the aforementioned methods based on statistical or machine learning achieved certain accuracy and application values, they generally relied on low-resolution time series hourly dataset that contains relatively little information and cannot benefit spike prediction. Moreover, statistical or machine learning models serve comparatively limited ability to learn nonlinear relationships within time series especially strong electricity price fluctuations. In contrast, forecasting skills using deep convolution neural networks (DCNN) [20–23] have been justified successfully in load forecasting for the short term and proved their predominant ability to learn discriminative features in nonlinear sequence analysis, which could be drawn spirits. Lago et al. [24] offered four different deep learning models to forecast electricity prices and demonstrated skills with deep neural networks achieving predominant accuracy rather than traditional statistical or machine learning ones. Deng et al. [25] devised a complicated structure of a deep neural network using dilated convolutional kernels and periodic coding to detect price spikes and capture severe price variations in market profiles, obtaining great improvements. Jahangir et al. [26] allocated proper bidirectional long short-term memory forecasting units to different shape clusters of electricity price series with K-means and Gaussian support vector machine. Hafeez et al. [27] designed a novel feature extraction process considering both entropy and mutual information, where candidate inputs are explored in order to cancel out the influences of unnecessary inputs based on the evaluation of their potential values. With elimination to fluctuation in electricity price, they used an LSTM model fed on extracted features to improve the forecasting accuracy. These recent works have proved the great potential of deep neural networks in electricity price forecasting and especially dealt with large fluctuation of prices appropriately. On the other hand, compared with single-step ahead electricity price forecasting, multistep prediction is more valuable in practice, like trading in the electricity market or scheduling BESS operations, which deep learning is skilled in.

However, the independent model cannot be effective for all cases, and each of them has its own advantages and disadvantages, especially for great variations in electricity price. For deep learning skills, their shortcomings mainly include local optimal solutions and hyperparameters setting, which bring unsatisfactory predictive performance. Great variances in electricity consumption and other exogenous factors lead to volatility and complexity within signal manifestation. Consequently, an independent forecasting model fed on an original single sequence of prices cannot superiorly express exact relationships. To address this issue, a combination of models with different mechanisms may have chances of price forecasting improvement depending on respective advantages [28]. Signal decomposition approaches like empirical mode decomposition (EMD), complementary ensemble empirical mode decomposition (CEEMD), variational mode decomposition (VMD), and singular spectrum analysis (SSA) have been utilized to explore more significant potential features located in the fluctuation of electricity price.

In general, researchers decomposed price series into several components, which are then delivered to respective forecasting units. The Sum of each component's prediction results is contributed to the final prediction. For California electricity and Brent crude oil short-term price prediction, Lahmiri [29] presented a VMD-based GRNN ensemble forecasting model. They used particle swarm optimization (PSO) to acquire GRNN hyperparameters. This hybrid model outperformed traditional algorithms based on machine learning and could be a promising methodology for price prediction. Qiu et al. [30] adopted EMD to decompose original electricity prices into several components called intrinsic mode functions (IMF). Then, advanced forecasting models are provided to extract tendencies for each IMF. At last, they gave a SVR model to incorporate all IMFs' prediction results and acquire an aggregated forecasting of electricity price. However, EMD has a disadvantage of end effect, which will cause negative impacts on decomposition accuracy. To improve this case, variants of EMD emerge continuously like ensemble empirical mode decomposition (EEMD) [31], fast ensemble empirical mode decomposition (FEEMD) [32], improved empirical mode decomposition (IEMD) [33], and improved complete ensemble empirical mode decomposition with adaptive noise (ICEEMDAN) [34]. A novel hybrid neural model based on EEMD and stochastic recurrent wavelet (SRW) was proposed [31], which enhances the precision and robustness of energy indexes price forecasting. Especially in their work, EEMD has proved a preferred means to deal with similar prices for decomposition. A hybrid evolutionary and adaptive models are developed by Jiang and Xuejiao [32] for electrical power system forecasting using the FEEMD approach, borrowing more strengths from a deep neural network. Zhang et al. [33] offered more complex mixture models including IEMD, ARIMA, and wavelet neural network (WNN), hyperparameters of which are also selected by fruit fly optimization algorithm. Their experiments showed that the decomposition strategy could benefit excellent feature extraction associated with load profiles. Another hybrid model relying on dual decomposition gained more attention [34], which overcomes the potential drawback of single-step decomposition in practice and brings more inspiration for electricity forecasting.

Although these popular hybrid models extracted significant features using EMD or extended EMD approaches, which gives forecasting models more strength, irregular nonstationary IMFs with high frequency as strong interference will affect the performance of the forecasting unit. Consequently, it is significant to handle nonstationary IMFs properly. In order to address this problem, we present a novel strategy of multiple nonstationary decomposition to decompose original electricity price signal into stable and significant components, which provides additional discriminative features to the deep neural network rather than EMD or extended EMD methods. Moreover, we devise a deep convolution neural network as a forecasting unit. Compared with the recurrent neural network, like LSTM and gate recurrent unit (GRU), it offers more powerful capability of learning nonlinear relationships in electricity price fluctuation and detection spikes instantaneously. Contributions of this paper are summarized as follows:

- We propose multiple nonstationary decompositions to extract the most significant components in price series, which express remarkably discriminative features in price fluctuation for regression prediction.
- Extracted components are fed into a devised deep convolution neural network with multiscale dilated kernels for multistep price forecasting. This structure could strengthen the ability to learn nonlinear relationships within electricity price fluctuation.
- More advanced price spike detection serves the optimized operation of battery energy storage system within Ontario grid connected microgrid. Sufficient experiments demonstrated that our proposed electricity price forecasting model provides excellent performances compared with the state-of-the-art approaches manifesting a promising prospect in economic benefits of operation in BESS.

Therefore, the main contribution of this paper is to propose a multiple nonstationary decomposition model for electricity price forecasting, which is used to optimize the operation scheduling of the battery energy storage system at the back of the meter. This paper focuses on two aspects, one focuses on the improvement of the price forecasting model, and the other tries to enhance economic savings of operation in BESS relying on deep recognition to the electricity price trends. This paper will be structured as follows: Section 2 introduces the key technologies and describes the details of our proposed method.  Section 3 introduces the experiment setups and discusses the performances of comparison experiments. Conclusions are given in Section 4.

## 2. Methodology

In this section, the operation of a BESS is described in detail considering an hour-ahead forecasting strategy. The components of our proposed electricity price forecasting model are then described.

### 2.1. Operation of BESS

When a BESS is being operated behind the meter, and MCPs are relatively lower, the power could be stored during this time to decrease local grid running costs. If the pressure of the grid grows during peak periods, the stored energy then could be delivered back to the local grid, reducing the necessary total electricity which will be bid from the wholesale electricity trading market at higher prices, which is able to improve profits of BESS owner. Besides, we do not consider some exogenous factors of BESS that would affect economic targets in our studies, such as cost of maintenance and investment loan interests. Our study tries to maximize the BESS operational economic profits with reasonable scheduling plans as follows:

(1) $$\begin{array}{c} \underset{l_{t}}{\max}E=\sum_{t=1}^{T}l_{t}{\overset{\wedge }{p}}_{t}\text{ subject to }\phi , \end{array}$$

where the objective equation (1) intends to enlarge the net savings with sophisticated operation approach, indicated by *E*. *T* expresses a fixed span of BESS scheduling unit, in our study *T*=24 for one-day-ahead planing. The unit of *l* is million watt (MW) and tells the charging/discharging behavior of BESS. In details, *l* is the total electricity to be discharged (*l*_*t*_ > 0) at time *t* for sales in local microgrid by charing (*l*_*t*_ < 0) from the electricity trading market. ${\overset{\wedge }{p}}_{t}$($/*MW*perhour) gives the electricity price prediction at time *t*. The target of equation (1) is to acquire the maximum under a set of constraints *ϕ* during operations of BESS, involving battery remaining capacity, rates of charging/discharging, emergency power for safety, etc. [35–37]. Our task mainly decides the charing or discharging amount of *l* at time *t*, and therefore in each step, the forecasting result of ${\overset{\wedge }{p}}_{t}$ plays a crucial role in BESS scheduling optimization problem with an aspect of economic savings.

In tradition, electricity market adopts day-ahead BESS operation strategy. According to historical price trends, utilities give the next day forecasting result and plan of scheduling horizon without any changes. Because of great variations in real-time electricity price, a day-ahead scheduling plan will result in large errors for electricity price forecasting, causing an economic loss of BESS business management. To alleviate great fluctuation on price forecasting, one feasible approach is called the rolling horizon model for BESS scheduling depending on updating price prediction one-hour-ahead, effectively in the microgrid system for economic management [38]. This model forecasts the next hour electricity price of each hour and tells if the price of the next hour is the spike during the current day. In fact, this procedure includes one-step and multistep predictions for spike detection. We suppose our scheduling plan applied in one day, *T*=24 in practice, and the scheduling horizon may be continuously changed over time. At 2:00 PM, operational scheduling plans are regularized dynamically in accordance with price predictions for the next 10 hours. Rolling horizon model predicts 3:00 PM and the remaining 9 hours electricity prices and judges whether 3:00 PM is a peak for the decision of BESS scheduling. Accordingly, when at 3:00 PM, the scheduling horizon contains the next 9 hours.

In recent years, high resolution dataset with 5 minutes MCPs has been applied in electricity price forecasting and optimization of BESS operation scheduling [11], which provides more information and benefits improvement of forecasting accuracy. With high resolution, great uncertainties of price fluctuation could be captured effectively and Chitsaz et al. [11] gave another approach of interhours rolling horizon (IRH). *γ* expresses the fraction of one hour for joining in current hour MCP forecasting. This hyperparameter can be customized according to user's requirement. For example, when *h*=10 and *γ*=5, IRH model uses first 5 MCPs to predict 10:00 AM MCP and five MCPs and its last 24 hours MCPs to predict 11:00 AM–24:00 PM MCP. On the union of a single step and multistep forecasting, IRH tries to detect whether 10:00 AM is located in the price spike in order to adjust operational scheduling of BESS in time for the economic target.

However, *γ* is a threshold designated by experience with higher sensitivity. The fixed constant *γ* will influence the performances of forecasting models in different areas or datasets. Besides, if *γ* is too large, new instructions of scheduling in BESS may not be carried out completely in the rest span of the current hour. In our previous work [25], an innovative operational scheduling approach of BESS is presented, allowing 5-minute MCPs forecasting no longer restricted to a complete hour but a span of 60 minutes between hours, as illustrated in Figure 1. Hyperparameter *γ* has been deprecated and the rolling window with 5-minute step is able to slide forward till the end of the day. In the study, we adopt our proposed strategy with devised forecasting model to optimize the operational scheduling of BESS.

### 2.2. EEMD

Nonstationarity is the most remarkable feature in electricity price series, generally manifesting great fluctuation and sharp peak, which gives serious difficulties to regression models. Researchers are attempting to disaggregate the original price sequence into significant and stationary components, setting up discriminative features to machine learning models or deep neural networks. Huang et al. published EMD for the first time, which tries to acquire an aggregation of IMFs and a residue signal approximating original one. As EMD holds a superior character of adaptiveness for nonlinear dataset analysis, it is extensively imported in various research fields [28]. EMD has some strong assumptions in order to obtain acceptable decomposition results:

1. Original signal contains at least two points with extreme values, including maximum and minimum values
2. Time scale in extreme points decides characters of initial signal in the local time domain
3. If there are only inflection points in the data without an extreme point, the extreme value is able to be acquired by differentiation strategy repeatedly to produce the final decomposition result by integration

In our study, the price dataset we used fits three assumptions and EMD should be effective theoretically. For a specific signal *X*(*t*), the procedure of process is as follows:

1. Search extreme points located in the original signal *X*(*t*)_*n*_
2. Cubic spline interpolation method is used to fit the lower envelope min(*t*)_*n*_ and the upper envelope max(*t*)_*n*_
3. Mean envelope ave(*t*)_*n*_=(min(*t*)_*n*_+max(*t*)_*n*_)/2, if ave(*t*) is close to 0, the iterative process terminates
4. *IMF*_*n*_=*X*(*t*)_*n*_ − ave(*t*)_*n*_
5. Let *X*(*t*)_*n*+1_=*X*(*t*)_*n*_ − *IMF*_*n*_ be a new original signal, repeat EMD decomposition process from (1)–(4)

EMD decomposition process is recursive through a screening process, repeating steps (1)-(4) for decomposition of the original sequence *X*(*t*)_*n*_. When the mean value *d*(*t*) is 0 or the stop criterion is satisfied, the iterative process is stopped. In each iteration, one *IMF*_*n*_ is generated, and the corresponding residual signal *X*(*t*)_*n*_ − *IMF*_*n*_ continues to be as a new original signal for decomposition. Through iterations precede, the number of extreme points is decreasing along with the generation of new IMFs that becomes intended significant components appropriating original *X*(*t*).

The phenomenon of mode mixing is a serious drawback of EMD decomposition, where one IMF consists of multiple signals with different frequency and amplitude. These IMFs are nonstationary and detrimental to forecasting models regardless of machine learning or deep neural networks. Moreover, nonstationary IMFs with different frequency or amplitude cannot reveal discriminative nonlinear relationships in the electricity price fluctuation of the trading market. Subsequently, Flandrin et al. [39] proposed EEMD method to solve the mode mixing problem. The model mixes white noise into initial series on the basis of the monotonicity of frequency distribution in stochastic noise. With the help of white noise, the stationary character of the original series is improved to a distinct extent, and the issue of mode mixing is effectively handled. Definitely, EEMD model is a striking breakthrough for optimization to EMD, and it works remarkably to improve the effectiveness and robustness of EMD. Meanwhile, other extended EMD like CEEMD methods continuously emerge that are dedicated to alleviating the influence of added white noise. However, in practice, EEMD and extended EMD still inevitably cause nonstationary IMFs with different frequency and amplitude. Signals with higher and unstable frequency are not suitable as hand-crafted features for forecasting models. As illustrated in Figure 2, the decomposition results hold obvious nonstationary IMF1-IMF4 components with higher frequency, which account for 50% of total IMFs and represent indispensable proportion of original signal information. If these remarkably nonstationary IMFs are completely ignored and no attention is paid to the forecasting model as some researchers did [40–42], the lost information undoubtedly hurts the accuracy of price forecasting, which gives large promotion space for service to deep learning models.

### 2.3. VMD

VMD is another extended signal decomposition approach with higher adaptiveness proposed in 2014 [43], which is able to disaggregate the electricity price series into several interesting modes. Completely nonrecursive and quasiorthogonal are remarkable qualities in VMD implementation. The effective strategy of variational mode is explored iteratively to identify the frequency center and bandwidth to each disaggregated mode. Equation (2) shows the variational problem of VMD.

(2) $$\begin{array}{c} \min_{\left(\eta_{k},\zeta_{k}\right)}\left\{\underset{k}{\sum }{\left\|\frac{\alpha }{\alpha_{t}}\left[\begin{array}{c} \psi \left(t\right)+\frac{j}{\pi } \end{array}\right]e^{j\zeta_{k}t}\right\|}_{2}^{2}\right\},\\ s\text{.t}.\;\underset{k}{\sum }\eta_{k}\left(t\right)=x. \end{array}$$

In equation (2), *η*_*k*_={*η*_1_, *η*_2_, *η*_3_,…, *η*_*K*_} represents the *K* modes obtained from the decomposition of VMD. *ζ*_*K*_={*ζ*_1_, *ζ*_2_, *ζ*_3_,…, *ζ*_*K*_} represents the frequency center of each mode. *x* expresses the input signal.

Two major parameters *k* and alpha of VMD have a great influence on the decomposition results, where alpha is the balancing parameter for VMD. The reasonable choice of these parameters can improve the effect of the decomposition so that the accuracy of prediction will be promoted.

The method envelope spectrum entropy (ESE) is used to select these two parameters. The entropy values of the signal decomposed by VMD are estimated by ESE. Initial values of *k* and alpha in decomposition are selected stochastically and the total entropy of all decomposed modes will be minimized. The calculation formula of entropy value is shown in the following equation:

(3) $$\begin{array}{c} Q_{nj}=-\sum_{t1=1}^{T}\frac{\beta_{t1}}{\sum_{t2}^{T}\beta_{t2}}\ln\left(\frac{\beta_{t1}}{\sum_{t2}^{T}\beta_{t2}}\right),\;j=1,2,\ldots ,k, \end{array}$$

where *β*_*t*1_ is the envelope spectrum of the signal *x* and the calculation expression is as follows:

(4) $$\begin{array}{c} \beta_{t1}=\sqrt{x^{2}+x^{\prime 2}}, \end{array}$$

where *x*′ with instantaneous value and phase angle are obtained by Hilbert transformation. Optimal *k* and alpha could be selected according to the results of sufficient experiments. In our study, *k* and alpha are set to 8 and 5, respectively. We tried to decompose nonstationary IMF1 and IMF2 with high frequency in Figure 2. Moreover, Figures 3 and 4 illustrate the results of the VMD decomposition. It is found that results of decomposition to IMF1 and IMF2 tend to be flat with relatively lower frequency, which is possible to be selected as additional hand-crafted features for forecasting models. Meanwhile, it addresses the issue of nonstationary IMFs that are not appropriately offered to price prediction, which would be borrowed from innovation spirit for electricity price prediction and optimization of operational scheduling in BESS.

### 2.4. TCMS-CNN Model

At present, most research has demonstrated electricity price forecasting models based on deep learning provide more superior performances rather than statistical and machine learning. Recent works using deep learning skills in majority focus on LSTM or GUR models [26, 27] and the deep convolutional neural network has already verified its excellent ability of nonlinear relationships extraction compared with RNN [20, 44, 45] in short-term load forecasting.

In the study, we optimize our previous work of multiscale convolutional neural networks using time-cognition (TCMS-CNN) for single and multistep short-term electricity price forecasting. The framework of our proposed model is illustrated in Figure 5.

TCMS-CNN model is a hybrid network of multiscale convolutional neural network and time-cognition models. In Figure 5, there are two subnetworks that constitute the entire network. The left subnetwork mainly consists of multiscale dilated convolutional layers, which provide different dilate ratios and serve the capability of learning local and global features. This mechanism benefits extracting complex nonlinear relationships in electricity price fluctuation. The right branch contains lots of fully connected layers that are fed on periodic coding of hours in each day and days in each week. Periodic coding stresses the uniqueness of the time period that offers more context exogenous features for deep analysis. In practice, we design coding styles relying on a unique markup of sin and cos functions. In the same way, the input of the left branch is a matrix divided into two parts, price vectors of each week filled in each row and corresponding periodic coding hours-week in a row of the other part. At the end of both branches, a feature fusion layer is provided for single or multistep electricity price forecasting. Temporal characters of the price series are extracted superiorly in our work, which provides an advanced prediction for optimization of operational scheduling in BESS.

### 2.5. Multiple Nonstationary Decompositions for Electricity Price Forecasting

Since electricity price reflects great variations and sharp peaks generally, some negligible IMFs produced by EEMD hold characters of higher and unstable frequency and amplitude, which expresses irregular features and affects the performance of a deep convolutional neural network for price forecasting. In this paper, we propose multiple nonstationary decomposition models with an end-to-end structure to optimize feature selection of signal decomposition that benefits the deep learning model for electricity forecasting.

In detail, as described in Figure 6, we adopt EEMD to decompose the original signal into *k* IMFs with different frequencies. *imf*1, *imf*2, *imf*3,…*imf*_*k*_ and res are obtained. In the next step, we need to select some IMFs that are unstable and should be processed further. There are some methods to define candidates. Our approach calculates the value of fuzzy information in each IMF and ranks them. Top 2 IMFs with large entropy could be chosen for further VMD decomposition. In fact, threshold 2 can be set as an experimental experience. Afterward, we use VMD to decompose these candidate IMFs into stationary and significant modes, acquiring *n* modes, respectively. Then, these products of EMD and VMD are together delivered to a sophisticated TCMS-CNN model for improvement of price forecasting accuracy. Sum of two branches prediction is the final price forecasting result. In another perspective, we understand this process as EEMD-VMD-CNN.

## 3. Case Study

### 3.1. Dataset Description

In this study, we evaluate the effectiveness and economic savings of our proposed models using Ontario's market electricity price dataset, where large consumers are referred to a peak demand over 50 kilowatts. IESO decides the wholesale price according to the relationship between buyers and suppliers in the real-time market, and bidding price is dynamically changing hourly [25].

In the union of Hourly Ontario Electric Price (HOEP), predispatch price (PDP) is generated as electricity price forecasting by IESO. IESO publishes PDPs in each hour for the next three hours on the website. Nevertheless, there is a clear inconformity between PDPs and HOEPs. Related deviation located in the year 2015 is around 38.49%, according to the definition (1/*n*)∑_*i*=1_^*n*^*abs*(*HOEP*_*i*_ − *PDP*_*i*_). If we intend to maximize the profits of BESS running, it is not advisable that decisions of operational scheduling are dependent on PDP, which cannot include sufficient information of price spikes. Consequently, it is necessary to devise an effective price forecasting model to provide accurate price prediction adaptive in the short and long terms. As shown in Figure 7, great fluctuation of nonstationary price series is remarkable and locations of the daily peak distribute stochastically in view. With a combination of short-long term price forecasting, IESO could simply give a conclusion if the current hour has attained the peak price in the trading market. The information of Market Clear Price, Ontario demand, total generation, etc., are included in the dataset. MCPs, which are set every five minutes, are used for single step prediction, and HOEP, a mean value of 12 MCPs in each hour, supports multistep prediction.

Some exogenous factors could be incorporated into electricity price short-term forecasting and scheduling of BESS models, involving weather, periodic information, and economic conditions [46]. Research has evaluated performances of several exogenous factors in the task of HOEP forecasting [47]. In our experiment, some electricity trading features including state load profiles, electricity consumption demand, generation magnitude, and flows are selected as inputs to devised models. In addition, other studies have reported an apparent influence of MCPs on price forecasting [11]. Therefore, we import historical MCPs into consideration for price short-term forecasting. To increase additional significant features of periodicity, sine-cosine encoding is also included as well.

At the beginning, in this dataset, small quantities of data are lost and redundant, and we restore the lost data by the nearest neighborhood interpolation and remove the redundant information. In addition, the dataset is divided into a training set, validation set, and testing set by 80%, 10%, 10%, respectively. Finally, the MCP in Ontario dataset is normalized into 0-1, which can reduce the error of the experimental results due to the drastic change of gradient.

### 3.2. Neural Network Training

Two subnetworks MS-CNN and fully connected networks, build up the baseline of our proposed model based on a multiscale deep convolutional neural network. The subnetwork on the left is MS-CNN, and the input data sequences contain historical load, holiday, and periodical coding. Subnetworks on the right hold two full connection layers, inputs of which are periodic encoding of many predicted steps. The representation vectors output from the two subnetworks are concatenated as inputs of the top-level fully connected layer for generating loads at the predicted steps. This framework ensures the model obtains sufficient characteristics, which enhances the understanding of the dataset. The parameters of our proposed model based on deep learning are shown in Table 1.

The training process of our proposed deep learning model is described in Figure 8, where after 20 epochs, the loss of target function will stay close to 0.00. Entire steady training denotes a better robustness complexity in deep learning computation, which implies excellent effectiveness of our proposed multiscale dilated convolutional neural network for electricity price forecasting. In experiments, the average time of forward inference is close to 0.02 seconds. All experiments were conducted on a cloud server with two NVIDIA P4 computing cards and the CPU with 8 cores. The implementations of machine learning tools are based on the StatsModels and scikit-learn packages, respectively. Other neural network-based models are realized by the Keras framework with Tensorflow backend.

### 3.3. Evaluation Metrics

This section evaluates the performance of electricity price forecasting from the perspective of statistics. Our forecasting model is trained on the dataset from the electricity market in Ontario, Canada, from 2012-2014 and tested on the data in 2015. The loss function of training adopts mean square error (MSE), and its calculation formula is as follows:

(5) $$\begin{array}{c} mse=\frac{1}{m}\sum_{i=1}^{m}{\left(y_{i}-{\overset{\wedge }{y}}_{i}\right)}^{2}, \end{array}$$

where *m* represents the total number of data samples, *y*_*i*_ denotes the ground truth, and ${\overset{\wedge }{y}}_{i}$ expresses the predicted values.

Mean absolute error (mae), root mean square error (*rmse*), and r-Square (*r*^2^) are used as evaluation metrics, and related formulas are defined as equations (6)–(8), respectively. The first two evaluation criteria are different description forms of error and a smaller value is preferred and reflects a better prediction result. In *r*^2^, the numerator part represents the sum of the square difference between real value and predicted value, and the denominator part tells the sum of the square difference between real value and mean value. The value range of *r*^2^ is [0,1]. If the result is 0, the model fitting effect is very poor; if the result equals 1, the model is error free. In general, a larger value *r*^2^ holds, the fitting effect is more acceptable. ${\bar{y}}_{i}$ denotes mean value of samples.

(6) $$\begin{array}{c} \text{mae}=\frac{1}{m}\sum_{i=1}^{m}\left|\left(y_{i}-{\overset{\wedge }{y}}_{i}\right)\right|, \end{array}$$

(7) $$\begin{array}{c} \text{rmse}=\sqrt{\frac{1}{m}\sum_{i=1}^{m}{\left(y_{i}-{\overset{\wedge }{y}}_{i}\right)}^{2}}, \end{array}$$

(8) $$\begin{array}{c} r^{2}=1-\frac{\sum_{i}{\left({\overset{\wedge }{y}}_{i}-y_{i}\right)}^{2}}{\sum_{i}{\left({\bar{y}}_{i}-y_{i}\right)}^{2}}. \end{array}$$

### 3.4. Statistical Analysis

In order to demonstrate the effectiveness of our proposed multiple nonstationary decomposition for electricity price forecasting, we use EEMD to decompose original electricity price series and prove the negative influence of IMFs with higher fuzzy information entropy on the performance of forecasting model. In practice, we choose multistep price prediction of 24 points for ablation study and a forecasting model based on ResNet. Experimental results are illustrated in Figure 9.

In the experiment, we acquired 8 IMFs and a res components which are delivered to the forecasting model, respectively, for 24 point prediction in a rolling manner. Then, with the same hyperparameters and white noise setting, the 24 points ground truth is (GT) also decomposed into 8 IMFs and res as GT. The difference between decomposed signals and GT is marked in red. It is easily found that IMF1 and IMF2 serve large distances because of their higher and different frequency, which reflects nonstationary EEMD IMFs will hurt the performance of price forecasting.

Therefore, in order to further improve the prediction accuracy, our proposed multiple nonstationary decomposition adopts VMD to decompose nonstationary IMFs. In our work, the threshold *k* is 2 and 2 IMFs is considered respectively further. All products from EMD or VMD are sent to TCMS-CNN for price forecasting respectively. The sum of all branches is the final prediction result. To verify the advantage of our proposed model EEMD-VMD-CNN, we compared it with the state-of-the-art works. TCMS-CNN has proved its great predominance in short-term load forecasting [20] and joined in our comparable study. Besides, a combination of EEMD and CNN models has been popular in the forecasting area providing attractive performances [48, 49], which is also selected as a subject for comparison called EEMD-CNN. Approaches based on VMD and CNN emerge recently as another focus in forecasting topic [50, 51] called VMD-CNN in this paper. For fairness in ablation study, the CNN model is TCMS-CNN and the dataset depends on Ontario's market electricity price dataset. Tables 2 and 3 show the single step and multistep of 24 hours prediction results of CNN, EEMD-CNN, VMD-CNN, and EEMD-VMD-CNN according to MSE, RMSE, MAE, and R2, respectively.

In Table 2, MSE, MAE, RMSE, and R2 of our proposed model EEMD-VMD-CNN are 0.1583, 0.0801, 0.3978, and 0.8632, respectively, in single step price forecasting. In 24 hours multistep prediction, the MSE, MAE, RMSE, and R2 of the hybrid model EEMD-VMD-CNN are 0.4865, 0.2424, 0.6975, and 0.5791. The prediction model EEMD-VMD-CNN proposed in this paper has the minimum MSE value, RMSE value, MAE value, and the maximum R2 value, which shows that the prediction effect of the model is remarkably superior. In addition, the performance of EEMD-CNN is more acceptable than VMD-CNN in both forecasting targets. VMD tries to extract features in another semantic space, and its experimental results imply the weakness of hand-craft feature discrimination. Price forecasting merely based on CNN is proved disadvantages obviously, since the amount of extracted significant features falls behind other hybrid models. Besides, accumulative errors lead to accurate prediction of a single step against multistep forecasting. Results of our ablation study demonstrate the predominance of our proposed approach that holds a promising prospect in electricity price forecasting.

In order to show the prediction ability of our proposed model more intuitively, the single step and multistep forecasting results of each model are plotted in comparison to the ground truth. As shown in Figures 10 and 11, the red line of the true price series can closely match the prediction curve and effectively capture its great fluctuations especially sharp spikes. It shows that the hybrid model EEMD-VMD-CNN proposed in this paper holds attractive prediction ability on single-step or multistep electricity price prediction.

In order to verify our proposed EEMD-VMD-CNN for single step or multistep electricity price forecasting, we imported another electricity price dataset collected from New South Wales (NSW) to evaluate the performance and quality of our proposed hybrid models. The experimental results are shown in Table 4, and it is found that our proposed model provides more competitive performances over MSE, MAE, RMSE, and R2 metrics. Although another dataset of electricity price dataset is tested for the study, EEMD-VMD-CNN served acceptable stable evaluations, which demonstrates better robustness rather than the state-of-the-art works. Specifically, the performances using the NSW dataset of our and other models were relatively mediocre than Ontario's as a result of different resolution in both datasets. Ontario's market electricity price dataset with 5 minutes MCPs contains great information to describe nonlinear relationships in price fluctuation. Nevertheless, the NSW dataset holds 30 minutes resolutions and is not good at reflecting sufficient potential rules in electricity price sequences.

### 3.5. Economic Analysis

We evaluate multiple nonstationary decomposition for electricity price forecasting from an economic perspective. Therefore, the electricity price forecasting relying on our hybrid model EEMD-VMD-CNN is applied in operations and dispatching of BESS in a local microgrid, Ontario, Canada. The microgrid plays a crucial role of a backup power supply when the main grid is cut off. The emergency power supply of the key load in the microgrid building should be provided by a 500 kW lithium-ion battery. Part of the battery capacity is required to reserve for emergency utilization. And rest capacity of storage could be utilized for energy trading to the main grid. In experiments, the capacity of the emergency load is defined as 150 kW. Battery's depth of discharge (DOD) runs around 70% and 200 kW can participate in the trading market.

According to the real-time electricity price change, the end-users in the power market can take corresponding measures to deal with the changes of electricity price at different times in each day in order to reduce their power operation cost [52]. Compared with the total load of the microgrid, the battery has a smaller volume, so any major power flow problems will not occur when the battery is running. The purpose of BESS scheduling optimization is to maximize profits. From another perspective, it is necessary to reduce the total amount of energy purchased from the electricity market in the peak period of high electricity prices. At the same time, the microgrid is injected from BESS in the price peak period because of the high price of electricity. In addition, nonprice factors such as renewable energy fluctuation or load balance may also affect the normal operation of the battery system in a microgrid. These factors should also be taken into account when operators formulate corresponding charging and discharging strategies. These factors have less influence and are not the focus of our research, and they are not considered here.

According to the electricity price forecast and historical data, in order to facilitate comparison, the following four charging and discharging strategies are considered:

1. Our proposed strategy: this model denotes our proposed multiple nonstationary decomposition for electricity price forecasting, illustrated in Figure 6, which adopts our presented TCMS-CNN that provides an excellent capacity of nonlinear relationships in price fluctuations. The multistep forecasting branch focuses on hour-level variations to predict rest hours price in one day, while the single-step branch pays more attention to five-minute resolution for the next 60 minutes forecasting. With both forecasting targets, it offers a reliable estimation for the detection of price spikes, which builds a solid foundation for the operational scheduling of BESS. The operation of the battery is determined by comparing the output of single step prediction and multistep prediction. When the current single step forecast price is higher than all subsequent multistep forecast prices, the battery will discharge in price spike, and vice versa.
2. PDP Scheduling: price forecasting via PDP public dataset. Nevertheless, these public datasets provide larger granularity with hour-level that serves limited information and cannot benefit optimization to operations of BESS scheduling.
3. Special strategy #1: mean price in hours calculated in 2003 and 2014, respectively, for supporting electricity price estimation. For acquiring the exact time of discharging, the candidate time is decided when the highest mean value comes, which is similar in decisions of charging.
4. Special strategy #2: whether discharging or charging is decided according to previous day experiences of price fluctuations.

In experiments, profits of comparative models are calculated each month, as shown in Figure 12. Through the difference between maximum and minimum of an entire day, the BESS scheduling is able to obtain up to $4553 of potential profits over the year 2015. Specifically, the decision of charging happens when the electricity price is located in the statistical lowest level in the dataset, and vice versa. In comparison, by applying our proposed multiple nonstationary decomposition model, 86.99% of the potential saving can be captured (totally $3960). The strategy of PDP scheduling holds the potential saving of 12.28% profit (total $559) only. Moreover, the special strategies #1 and #2 give 39.26% and 26.99% (totally $1787 and $1229), respectively. As PDP scheduling lives only on an hourly resolution dataset, the profit margin is relatively lower, which demonstrates the effectiveness of our hybrid model with fine-grained resolution. These statistical results reflect the remarkable performance of our proposed electricity forecasting model.

Our strategy has the highest economic benefit in every month, and February is the best.

Table 5 shows the percentage of each strategy over 12 months in year 2015 relative to the possible maximum profits. Statistically, our proposed multiple nonstationary decomposition model outperformed others in each month and reached the highest income of 95.069 5% ($740 in total, $779 in expectation) in February. Compared with other methods, our proposed approach can increase the revenue by 43.270 7% maximum and 25.542 4% minimum, respectively, at least. The model based on PDP scheduling provides unacceptable performances because of low-resolution dataset that cannot provide more valuable information. Both special strategy #1 and special strategy #2 have similar average performances but distinct in each month. They are determined by statistical experience and not convincing as a result of changes in microgrid structure and behaviors of end-users. Only one-hour-ahead forecasting could grasp real-time trends in the electricity market.

## 4. Conclusion

With emerging of hybrid models with signal decomposition, popular methods like EMD and extended EMD approaches cannot address the issue of nonstationary decomposed components, which has a negative influence on the performance of the forecasting unit. In this paper, we propose an innovative electricity price forecasting model for the optimization of operational scheduling in BESS from an economic perspective. At first, we use EEMD to acquire IMFs from the original price series. In addition to nonstationary components with higher frequency and different amplitudes, VMD is adopted to process them and produce more stable modes. Moreover, all products from EEMD and VMD are fed to our devised multiscale and time recognition convolutional neural network for price forecasting, respectively. Results of all branches are summed up as the final prediction. In comparison to the state-of-the-art methods, our presented approach reflects remarkable superior performances, which strengthens optimization of scheduling in BESS for the purpose of economic profits. Through sufficient economic analysis, in comparison to another scheduling strategy, our method obtains the largest profit savings obviously, which manifests a promising prospect in the electricity market.

There is a strong assumption that our BESS serves a smaller capacity compared with the whole trading market, which cannot influence the bidding prices and can be operated without consideration of market factors. In contrast, if the scale of BESS becomes larger, the influence of operations should be taken into account. Besides costs of equipment maintenance and depreciation, investment interests are not considered in our work that should not be ignored in practice.

Future works contain designing more advanced multitask deep learning network to improve performances of price forecasting and spike detection, which should be adaptive in different electricity market using transfer learning skills, in order to enhance generalization and robustness of our work. Furthermore, online learning should be studied to promote the practicality of electricity forecasting models.

## Figures and Tables

**Figure 1:** Our proposed ITRH framework. We adopt this strategy with a well-established electricity forecasting model to optimize the operational scheduling of BESS.

**Figure 2:** Results of the EEMD decomposition. IMF1-IMF4 shows great nonstationary components. Res denotes the trend of the original signal.

**Figure 3:** Results of VMD decomposition for IMF1 from EMD decomposition.

**Figure 4:** Results of VMD decomposition for IMF2 from EMD decomposition.

**Figure 5:** Two subnetworks MS-CNN and fully connected networks constitute the backbone of TCMS-CNN. At the end of two branches, a fully connected layer fuses features extracted from a multiscale dilated neural network and periodic coding model. This design ensures an excellent ability to learn nonlinear relationships in electricity price fluctuations.

**Figure 6:** Framework of our proposed electricity price forecasting with an end-to-end structure. The original price series is first decomposed using EEMD. According to fuzzy information entropy, two nonstationary components are selected to be decomposed by VMD furthermore. A different group of significant components is sent to the TCMS-CNN model for price forecasting respectively. Both results of branches are added as the final price prediction.

**Figure 7:** Illustration of electricity price fluctuation.

**Figure 8:** Training process of our proposed model based on deep learning for price forecasting.

**Figure 9:** Forecasting results of each IMFs and res by EEMD, which shows nonstationary IMFs, affect the performances of electricity price forecasting and significance of our proposed multiple nonstationary decompositions.

**Figure 10:** The result of single-step prediction. The horizontal axis represents a different time, the vertical axis is electricity price, the black line denotes real electricity price data, and the red line is EEMD-VMD-CNN prediction. The predicted and the real curve closely fit each other.

**Figure 11:** The result of 24-hour multistep prediction. Compared with single-step prediction, the predicted value curve has a relatively weak fitting effect because of accumulative errors within the rolling process, but it can also capture most of the peak points.

**Figure 12:** Monthly economic benefits of each model.

**Table 1:** Shared parameters of neural network models and related strategies selected.

Parameters	MS-CNN
Depth	34
Hidden neural	None
Kernel size	8
Kernel number	24
Batch size	128
Input length	336
Dropout rate	0.05
Loss function	MSE
Optimizing method	AMSGrad
Start learning rate	0.01
Learning rate decay	0.3
Training stop	Early stopping

**Table 2:** Comparison results of CNN, EEMD-CNN, VMD-CNN, and EEMD-VMD-CNN models for single step electricity price forecasting.

Model	CNN	EEMD-CNN	VMD-CNN	EEMD-VMD-CNN
MSE	1.8735	0.4831	0.6453	**0.1583**
MAE	0.2578	0.1097	0.1846	**0.0801**
RMSE	1.3687	0.6951	0.8033	**0.3978**
R2	0.3067	0.6098	0.5763	**0.8632**

**Table 3:** Comparison results of CNN, EEMD-CNN, VMD-CNN, and EEMD-VMD-CNN models for multistep electricity price forecasting of 24 hours.

Model	CNN	EEMD-CNN	VMD-CNN	EEMD-VMD-CNN
MSE	3.1262	0.7667	0.9779	**0.486 5**
MAE	0.8976	0.5097	0.5764	**0.242 4**
RMSE	1.7681	0.8756	0.9889	**0.6975**
R2	0.1023	0.4034	0.3476	**0.5791**

**Table 4:** Comparison results of CNN, EEMD-CNN, VMD-CNN, and EEMD-VMD-CNN models for single step electricity price forecasting using NSW dataset.

Model	CNN	EEMD-CNN	VMD-CNN	EEMD-VMD-CNN
MSE	4.363	1.281 7	1.008 9	**0.585**
MAE	1.581	0.956 2	0.69	**0.273 4**
RMSE	2.901 8	1.727 3	1.318 8	**0.743 6**
R2	0.205 6	0.473 5	0.451 6	**0.772 5**

**Table 5:** The percentage of each strategy over 12 months in the year 2015 relative to the ideal maximum profit (%).

	Our proposed	PDP	Special	Special
	Nonstationary decomposition	Scheduling	Strategy #1	Strategy #2
Jan.	81.837 6	**51.798 8**	11.660 5	7.374 4
Feb.	**95.069 5**	8.163 9	29.213 6	12.116 5
Mar.	88.411 2	8.156 3	67.714 5	45.967 6
Apr.	86.453 6	10.294 6	55.565 7	22.988 7
May.	91.755 7	0.897 9	23.898 0	11.639 3
Jun.	90.357 5	2.620 7	31.324 6	**52.630 4**
Jul.	78.803 4	12.622 1	55.212 5	41.011 6
Aug.	93.958 4	3.589 2	36.566 3	31.644 1
Sep.	86.154 4	22.893 0	43.569 6	39.539 0
Oct.	50.663 1	4.123 6	37.451 0	17.173 7
Nov.	92.006 3	13.672 6	**69.527 1**	43.549 1
Dec.	88.009 7	17.420 9	35.776 5	40.690 3
Average	85.29	12.946 3	41.456 7	30.527

## Data Availability

The raw data supporting the conclusions of this article will be made available by the authors without undue reservation.
